RETRACTED

# Effect Evaluation of Artificial Intelligence-Based Electronic Health PDCA Nursing Model in the Treatment of Mycoplasma Pneumonia in Children

**DOI:** 10.1155/2022/1956944

**Published:** 2022-03-11

**Authors:** Yan Zhao

**Affiliations:** Department of Pediatrics in Affiliated Hospital, North Sichuan Medical College, Nanchong 637000, Sichuan, China

## Abstract

The PDCA cycle, also known as Deming's cycle, mainly includes four stages: planning, implementation, inspection, and processing. As a kind of atypical pneumonia with fever and cough, mycoplasma pneumonia harms the health of many children. The purpose of this study is to investigate the anti-inflammatory and antimycoplasma effects and safety of artificial intelligence e-health PDCA nursing mode on pediatric MPP, to investigate its clinical efficacy, to observe the changes of serum cytokines (IL-10, IL-2, IL-4, IFN-*γ*), and to explore the mechanism of action and possible targets for the treatment of MPP, to provide a new basis for clinical treatment of MPP. The experimental results show that in the experimental group using PDCA nursing mode, the total satisfaction is 97.22%, higher than the control group of 94.44%; in the experimental group, the hospital stay and symptom disappearance time were significantly shortened by four hours. The satisfaction of nursing staff was significantly increased in statistical significance (*P* < 0.05). Therefore, in a statistical sense, the artificial intelligence e-health PDCA nursing mode can significantly improve the clinical symptoms of MPP children with wind-heat stagnation of lung syndrome and phlegm-heat closure of lung syndrome, improve the treatment effect of childhood mycoplasma pneumonia epidemic, shorten the time of hospitalization and symptom disappeared, and play a great auxiliary role in the treatment of childhood mycoplasma pneumonia.

## 1. Introduction

### 1.1. Research Background

Mycoplasma pneumonia (MPP) is a kind of atypical pneumonia with fever, severe irritant dry cough, and mild pulmonary signs. The main cause of the disease is the infection of pathogenic mycoplasma *pneumoniae* (MP). In recent years, studies have shown that the incidence of MPP has increased significantly, and it is even the primary pathogen in some age stages, accounting for about 30% of CAP, and the onset age tends to be younger. With the widespread use of antibiotics, the drug resistance rate of MP varies from 3.6% to 36.4%, showing an increasing trend. The drug resistance rate of MPP children varies greatly in specific regions due to the influence of regional, climate, and other factors. Some studies showed that in vitro drug resistance experiments were as high as 90–100%, suggesting that the situation of MP drug resistance was very serious. In addition, the long-term and widespread application of antibiotics is prone to various problems such as drug resistance of superbacteria, loss of regulation of bacterial community, and double opportunistic infection. Therefore, how to improve the clinical efficacy and safety of drug treatment of MPP and reduce the drug resistance rate has become the difficulty of clinical breakthrough.

RETRACTED

The clinical manifestations of “pneumonia cough” are mainly “heat, cough, phlegm, wheeze, and panting.” The external cause is that the external evil invades the lungs, and the lungs lose their function of sending out and descending. Internal causes are mainly responsible for the weakness of children's viscera, Yin and Yang and juvenile organs, the imbalance of strength and weakness of the five viscera, and the fragile and unstable correlation, and the evil spirit is easy to be committed by the guest; or the righteous qi in the body is weak, the function of the spleen and stomach is low, and it is easy to be infected with evil qi. The fundamental treatment lies in syndrome differentiation and treatment. Different syndromes and treatment methods are different. With the development of this disease, modern TCM experts, based on their practical experience in diagnosis and treatment, have carried out syndrome differentiation and treatment on MPP from different perspectives, so as to fully explore the great advantages of TCM in China.

Artificial intelligence is a new technical science that studies and develops theories, methods, technologies, and application systems for simulating, extending, and expanding human intelligence. Artificial intelligence is a branch of computer science that attempts to understand the essence of intelligence and produce a new type of intelligent machine that responds in a similar way to human intelligence.

The name of PDCA comes from the initials of the English words Plan, Do, Check, Act, also known as the improvement cycle. The methodology describes the four steps of the system to achieve continuous improvement and defines our continuous approach to improving product and process quality. The introduction of PDCA management mode in medical treatment will be a more efficient cooperation mode for hospitals, patients, and medical staff.

### 1.2. Research Status at Home and Abroad

At home and abroad related to electronic health, the PDCA mode of nursing research, and child mycoplasma pneumonia, Lin WC sees that artificial intelligence (AI) technology provides a promising approach for the analysis of electronic health records more modal datasets, such as to provide an overview of different methods of artificial intelligence applied to the electronic medical record data in the field of ophthalmology. Although AI technology has been widely used in imaging data, studies using AI technology for clinical data from electronic medical records are limited [1]. SUBBA enables real-time monitoring and intervention in healthcare. Electronic health records (EHRs), mandatory in the most developed countries, can use evidence-based tools to help make safer decisions about patient care. However, there are few examples applied to the PDCA nursing model [2]. Wang K used transcriptome sequencing to identify gene expression and selective splicing profiles to gain insight into the pathogenesis of severe MPP. Bronchoalveolar lavage fluid (BALF) samples from 3 children with severe MPP and 3 children with mild MPP were deeply sequentially analyzed, calculated and annotated, and quantitatively analyzed. Gene expression analysis showed that compared with mild MPP, children with severe MPP had 14 upregulated genes and 34 downregulated genes, but there was a need to improve the nursing model to improve it [3]. In management, the PDCA cycle management model is a general management model, which has been widely used in hospital nursing quality management in recent years. Through the effective application of this management model, the work efficiency of nursing staff can be continuously improved.

RETRACTED

### 1.3. Main Innovation

Routine nursing often appears normative and has a lack of planning and other problems, resulting in the reduction of the effect of medical adjuvant treatment and slow recovery of patients, and nursing adverse events also occur frequently. In this article, PDCA nursing mode was added in the treatment process of chlamydia pneumonia in children to increase effective nursing intervention. A comparative analysis was conducted from multiple perspectives, such as the length of stay between the experimental group and the control group. It can be seen that PDCA nursing can alleviate the symptoms of children, improve the satisfaction of patients and nursing staff, shorten the length of hospital stay and symptom disappearance time, and reduce nursing adverse events. PDCA nursing mode changes the retrospective case analysis method adopted by traditional management through continuous quality improvement. It carries out three-level ward rounds or nursing rounds for difficult cases or cases that need assistance from the superior in nursing. The form of PDCA can be 1–2 times a month and can be used to improve nursing operations and procedures. The basic principle of its operation is that everything needs to be planned in advance, so that the nursing process is orderly, reduce the occurrence of repeated nursing, excessive nursing, omission nursing, and so on. This article innovatively introduced PDCA nursing mode in the treatment of children with mycoplasma pneumonia and added the wavelet transform theory of artificial intelligence to make the whole nursing mode intelligent.

RETRACTED

## 2. Proposed Method

Wavelet transform has a better effect on nursing mode management and is one of the key research directions of researchers now. The core idea of wavelet analysis is as follows: firstly, the wavelet is stretched and shifted, and then, the correlation between the image and the wavelet is studied. In fact, the wavelet is a function, which fluctuates in the local area.

### 2.1. Principle of Wavelet Transform

In a broad sense, intelligent robot refers to the humanoid or other forms of artificial machines with some human abilities. It is generally believed that intelligent robot should have perception ability, planning ability, movement ability, and coordination ability. Although the intelligence level of the robots developed at present is still not very high and there is still a big gap between them and the real-life intelligence, at present, rich achievements have been made in the research of intelligent robots at home and abroad, and they continue to penetrate into all fields of human activities [4, 5]. On the basis of existing technology, people customize various types of robots according to the actual needs of all walks of life for detection, disaster relief, transportation, delivery, cleaning, etc., and these robots can replace people to accomplish some high-risk, monotonous work, to a great extent, the human liberation, causes humans to do more creative work and improve the social productivity.

### 2.2. One-Dimensional Wavelet Transform Algorithm

In some commonly used signal analysis methods, Fourier transform is a kind of analysis method that researchers like to use very much. However, Fourier transform is a pure frequency-domain method, so frequency information in local time period cannot be obtained [6, 7]. Although STFT can be used to analyze the characteristics of signals in the time domain and the frequency domain at the same time, it is not conducive to analyzing pulse signals because of the fixed time window. Wavelet transform is a new theory deduced based on Fourier transform. Compared with Fourier transform, wavelet transform is a time-frequency multiresolution analysis method starting from local angle [8, 9].

The function *ϕ*(*t*) satisfies the following admissibility conditions:

(1) $$\begin{array}{c} C_{\phi }=\int_{-\infty }^{\mathrm{+\infty}}{\left|\omega \right|}_{\left|\psi \left(\omega \right)\right|}d\omega \;<\infty , \end{array}$$

where *ψ*(*t*) is the parent wavelet and *ψ*(*ω*) is the Fourier transform of *ψ*(*t*). After multiple stretching and translation operations on the parent wavelet, the family of wavelet functions *ψ*_*m*,*n*_(*t*) can be obtained as follows [10, 11]:

(2) $$\begin{array}{c} \psi_{m,n}\left(t\right)=\frac{1}{\sqrt{m}}\psi \left(t-n\right), \end{array}$$

where *m* is the scale factor and *n* is the displacement factor.

RETRACTED

Discrete wavelet analysis is adopted in this article, and the discrete wavelet *ψ*_*s*,*w*_(*t*) is defined as follows [12]:

(3) $$\begin{array}{c} \psi_{s,w}\left(t\right)=\frac{1}{\sqrt{m_{0}^{w}}}\psi \left(t-qn_{0}m_{0}^{w}\right), \end{array}$$

where s and w are integers, m_0_ is an integer greater than 1, and *n*_0_ is a constant greater than zero. The discrete wavelet transform of the function *f*(*t*) is [13]

(4) $$\begin{array}{c} WT_{f}\left(s,w\right)=<f\left(t\right),\psi_{s,w}\left(t\right)>=\int_{-\infty }^{+\infty }f\left(t\right)\bar{\psi_{s,w}\left(t\right)}dt, \end{array}$$

where 〈〉 denotes the inner product and $\bar{\psi_{s,w}\left(t\right)}$ denotes the complex conjugate of *ψ*_*s*,*w*_(*t*). Direct use of a low-pass filter may lose the contour feature information of the signal, and direct use of a high-pass filter may retain a lot of interference components, so only two filtering methods cannot be directly selected in pulse signal processing. Although the signal waveform after Fourier transform denoising will become relatively smooth, it will lose a lot of details. The use of wavelet transform can overcome the above contradictions and has a significant advantage in the study of the detailed characteristics of signals [14, 15].

Generally speaking, the wavelet coefficient of noise is small. When the coefficient is less than a certain set threshold, this part can be treated as caused by noise and all of it can be set to zero. When the value is greater than the set threshold, it can be considered that it is mainly caused by useful signals, and it can be kept unchanged, or it can be contracted by a fixed amount as shown in following the formula [16, 17]:

(5) $$\begin{array}{c} {\hat{\omega }}_{j,k}=\left\{\begin{array}{c} \omega_{j,k},\left|\omega_{j,k}\right|\geq \lambda \\ 0,\left|\omega_{j,k}\right|<\lambda \end{array}\right.,\\ {\hat{\omega }}_{j,k}=\left\{\begin{array}{c} sign\left(\omega_{j,k}\right)\left(\left|\omega_{j,k}\right|-\lambda \right),\left|\omega_{j,k}\right|\geq \lambda \\ 0,\left|\omega_{j,k}\right|<\lambda \end{array}.\right.. \end{array}$$

In the new threshold function, the part less than *λ* is still treated in the same way as the method mentioned above; the part greater than *λ* is treated by combining two classical functions with variable *μ*, under the limit condition *μ*⟶0 and the part greater than *λ* is treated as a hard threshold function. When the limit condition *μ*⟶1 is satisfied, the improved soft threshold function is used for the part greater than *λ*. The new threshold function is shown in the following formula [18, 19]:

(6) $$\begin{array}{c} {\hat{\omega }}_{j,k}=\left\{\begin{array}{c} \left(1-\mu \right)\omega_{j,k}+sign\left(\omega_{j,k}\right)\left(\left|\omega_{j,k}\right|-\exp\left(\lambda -1\right),\left|\omega_{j,k}\right|\right.\geq \lambda \\ 0,\left|\omega_{j,k}\right|<\lambda \end{array}.\right.. \end{array}$$

According to the formula, the improvement of the new threshold function lies in that, and the part of |*w*_*j*,*k*_| ≥ *λ* is replaced by the content shown in the above formula and retained as the new wavelet coefficient. The basic idea of the improved method is derived from the weighted average combination of soft and hard threshold functions. It not only has the advantages of the two methods but also overcomes their respective shortcomings. Compared with the traditional hard and soft threshold functions, the new threshold function has higher reconstruction accuracy and better denoising effect. In addition, the traditional soft threshold function has the problem of discontinuous derivative, while the new threshold function is continuous derivative, which is more convenient in dealing with other kinds of mathematical problems and has a wider range of practical application, so it has obvious advantages. Therefore, this article uses the method after the improved threshold function to realize the denoising of pulse signal [20].

RETRACTED

When the wavelet energy is used as the eigenvector of the pulse category, the rate of the pulse recognition process may be affected due to the large number of wavelet scale division and the larger dimension of the eigenvector. Principal component analysis (PCA) technology can reduce the loss and can be used to simplify the pulse feature vector, obtain the principal component feature parameters with less dimension, and it can show almost all information, which can improve the system identification efficiency. The process of reducing the dimension of pulse signal feature vector *E* by using principal component analysis technique is as follows:

(1) The *m* n-dimensional eigenvectors *E* obtained are written into a dimensional data matrix *n* × *m*. The matrix *E* is normalized according to the following formula, and the normalized matrix is obtained to eliminate the interference of data dimension:
  (7) $$\begin{array}{c} E_{ij}^{*}=E_{ij}-{\bar{E}}_{i}, \end{array}$$
where $\bar{E_{i}}$ is the sample mean and *s*_*i*_ is the sample standard deviation.
(2) Calculate the covariance matrix *E*^*∗*^ of the normalized matrix according to the following formula:
  (8) $$\begin{array}{c} \overset{1}{\underset{m-1}{c=}}\sum_{j-1}^{m}\left(E_{ij}^{*}\right.-\bar{\left.E_{i}^{*}\right)}\left(E_{ji}^{*}-\bar{E_{j}^{*}}\right)\overset{1}{\underset{m-1}{=}}E^{*}E^{*T}, \end{array}$$
(3) Calculate the eigenvalues of C and their eigenvectors, adjust the corresponding eigenvectors according to the eigenvalues, and obtain the unit orthogonal matrix according to the Schmidt algorithm.
(4) Calculate the cumulative contribution rate of eigenvalues, set the extraction index as *η*, and get the number of main elements *k* and corresponding main vectors *V*^*∗*^ that meet the requirements.
(5) Calculate the projection of the normalized matrix *E*^*∗*^ on the main vector *X*=(*x*_*ij*_)_*k*×*m*_, and obtain the low-dimensional eigenvector *X*=[*X*_1_, *X*_2_,…, *X*_*k*_] according to the following formula:
  (9) $$\begin{array}{c} X=V^{*T}E^{*}. \end{array}$$

In this article, the eigenvalue, contribution rate, and cumulative contribution rate of each component of the 8-dimensional eigenvector obtained from the wavelet energy are shown in Table 1.

RETRACTED

### 2.3. Two-Dimensional Wavelet Transform Algorithm

Simply put, the one-dimensional wavelet is extended to the two-dimensional wavelet, and the one-dimensional wavelet transform is equivalent to the two-dimensional wavelet transform when the two-dimensional image data are carried out independently in the horizontal and vertical directions:

(10) $$\begin{array}{c} W_{f}\left(a,b_{x},b_{y}\right)=\iint f\left(x,y\right)\psi_{a,b_{x},b_{y}}\left(x,y\right)dxdy, \end{array}$$

where *b*_*x*_ and *b*_*y*_ represent the translation on two dimensions, *a* represents the scale factor, *f*(*x*, *y*) ∈ *L*_2_(*R*) is a two-dimensional arbitrary function, and *W*_*f*_(*a*, *b*_*x*_, *b*_*y*_) is a two-dimensional wavelet transform coefficient.

The inverse transform of two-dimensional wavelet transform is

(11) $$\begin{array}{c} f\left(x,y\right)=\frac{1}{c_{\psi }}∭w_{f}\left(a,b_{x},b_{y}\right)\bar{\psi_{a,bx,by}}dxdy. \end{array}$$

Under the action of the same principle, the above theoretical methods can be pushed to higher dimensions. The two-dimensional wavelet transform is to carry out the discrete transform on the image, and carry out the multiscale decomposition and reconstruction of the wavelet based on the obtained discrete transform:

Let *W*_*j*_ be the closure on the set {*ϕ*_*jk*_(*t*); *k* ∈ *Z*} linearly spanned, and then

(12) $$\begin{array}{c} L^{2}\left(R\right)=\cdots ⊕W_{j-1}⊕W_{j}⊕W_{j+1}⊕\cdots . \end{array}$$

Yeah, there is a unique solution to *f*(*t*) ∈ *L*^2^(*R*):

(13) $$\begin{array}{c} f\left(t\right)=\cdots +g_{-1}\left(t\right)+g_{0}\left(t\right)+g_{1}\left(t\right)+\cdots . \end{array}$$

One of *g*(*t*) ∈ *W*_*k*_, *k* ∈ *Z*. For each *k*, let us think about it：

(14) $$\begin{array}{c} V_{k}=\cdots +W_{k-2}+W_{k-1},k\in Z. \end{array}$$

Each *V*_*k*_ is the set of all the displacements *ϕ*_*jk*_(*t*) containing the scale ≤*k* − 1.

RETRACTED

Wavelet reconstruction is the inverse process of wavelet decomposition. Reconstruction is to synthesize the multiscale wavelet into the original signal source by using the wavelet coefficient under the multiresolution obtained by wavelet decomposition. Reconstruction is not completed immediately after decomposition, which can complete the process of image defogging and so on.

The application of wavelet transform to image processing mainly has the following advantages:

1. Wavelet transform can cover the whole part of the image.
2. The wavelet transform theory is to use the filter that selects the image suitable, so that the correlation between different features of the information extracted from the image can be reduced or removed to the maximum extent.
3. The theory of wavelet transform has the characteristics of frequency conversion. High frequency resolution and low time resolution can be used in the low frequency part of the image, and low frequency resolution and high time resolution can be used in the high frequency part of the image.
4. Fast algorithm can be used in the actual operation of wavelet transform; that is, Mallat wavelet decomposition method is often used.

Because of these advantages of the wavelet transform, this article uses the wavelet transform method and will further analyze the wavelet transform in the following description.

### 2.4. PDCA Nursing Model

PDCA cycle is a continuous spiraling cycle rising process, which can be divided into four stages and eight steps, and each stage is gradual in order to promote the improvement of project quality.

The first is the quality management planning stage: the task of this stage is mainly to determine the quality objectives of the project, formulate implementation plans, and plan management measures. It can be roughly divided into four specific steps: 1. study the status quo of the project and find out the quality defects of the project. 2. Analyze the causes of project quality defects and all influencing factors. 3. Find out the main reasons and factors that cause quality problems. 4. For the results of the previous step, make targeted quality improvement measures, and determine the expected goals and detailed implementation plans.

RETRACTED

PDCA can be divided into four stages. The first stage is, P stage, the planning stage. In this stage, in order to form a certain planning scheme, an enterprise needs to clarify its performance objectives and then further determine relevant performance appraisal indicators through top-level design, planning, and inspection. The second stage, stage *D*, is the execution stage. This stage is to carry out the plan formed in the planning stage, and all the work will be carried out in an orderly manner according to the plan. The third stage—stage C, is the feedback stage. This stage is to analyze and feedback the implementation effect of the implementation stage, to monitor the progress, to check the original plan, and to find out the situation beyond the plan and point out the deficiencies. The fourth stage—A stage, is the improvement stage. This stage is to reflect on the problems found in the third stage, acknowledge or deny, and advantages need to be further developed, and deficiencies need to summarize experience and to improve efficiency.

PDCA has the following characteristics: first, a large ring set small ring. The PDCA cycle is a large cycle with a smaller PDCA cycle. The smaller level PDCA cycle is formulated according to the larger level PDCA cycle. The larger level PDCA cycle plays its role thanks to the effective execution of the smaller level PDCA cycle, recurrent relationship.

Second, keep improving and rising. PDCA will solve some problems and accumulate new experience every time it completes a cycle. A large number of problems will be improved and improved in the cycle process. New goals and contents will also appear in each cycle, so as to improve the management level of enterprises and achieve the development of enterprises.

Third, pay attention to the A cycle. In the PDCA cycle, stage A, the improvement stage, is the key. Stage A is the process of improving the problems found in the previous three stages, and it is the key step from quantitative change to qualitative change. Only by improving the problems found can we constantly push things forward. If there is no improvement stage, then things cannot be completed and improved, only the same, so stage A is a key link to promote the development of things.

In view of the above advantages, this article innovatively applied the PDCA cycle mode in the treatment of mycoplasma pneumonia in children.

### 2.5. Support Vector Machine Method Based on Machine Learning

In recent years, with the development of science and technology, people gradually use intelligent computers to replace some tedious manual labor and mental labor, and have achieved remarkable results. For example, using computers to recognize human speech by learning, learn checkers, detect rare diseases, detect credit card fraud problems, driverless cars, etc. These are achieved through the intelligent learning of the computer. Machine learning is one of the important frontier disciplines that combine computer science and information science.

RETRACTED

The simplest classification model in SVM is the maximum margin classifier W. In a linear classification problem, define a linear function for

(15) $$\begin{array}{c} g\left(a\right)=w^{T}a+b, \end{array}$$

where a is the vector representation of the sample data, and the dimension can be very high. Assuming that the threshold is 0, the category to which the sample a belongs is determined according to the positive or negative of the *g*(*a*) value.

In order to maximize the target geometric interval, it can be transformed to solve the following optimization problem as

(16) $$\begin{array}{c} F=\min\frac{1}{2}{\left\|w\right\|}^{2}. \end{array}$$

The maximum geometric interval is achieved here, where ‖*w*‖^2^ is a parameter that controls the classification surface. Using the Lagrangian function to derive the dual form of the above optimization problem is

(17) $$\begin{array}{c} L=\sum_{\mathrm{i=1}}^{n}\alpha_{i}-\frac{1}{2}\left|\sum_{\mathrm{i,j=1}}^{n}\alpha_{i}\alpha_{j}b_{i}b_{j}\right|, \end{array}$$

where the Lagrangian coefficient *α*_*i*_ is the solution of the optimization problem.

Since many data in the real world are noisy, the feature space generally cannot be separated. In order to balance model performance and generalization, slack variables are introduced, which can allow a small number of error points and outliers. The optimization problem is finally transformed into the following:

(18) $$\begin{array}{c} F=\min\frac{1}{2}{\left\|w\right\|}^{2}+C\sum_{i=1}^{n}\xi_{i}. \end{array}$$

The measurement of the expiratory flow rate is an index that mainly reflects the degree of obstruction of the large airway. It is more sensitive and objective than clinical symptoms to reflect the degree of airway obstruction and changes in the condition of asthma patients. Monitoring expiratory flow rate can help detect early signs of disease deterioration before symptoms appear, where C is the penalty coefficient. Similarly, using the Lagrange multiplier method, the above optimization problem is transformed into the following dual problem as

(19) $$\begin{array}{c} L=\sum_{\mathrm{i=1}}^{n}\alpha_{i}-\frac{1}{2}\left(\sum_{\mathrm{i,j-1}}^{n}\alpha_{i}\alpha_{j}b_{i}b_{j}a_{i}^{T}\right). \end{array}$$

Solve the above problem, solve the coefficient *α*_*i*_, and get the optimal classification plane. The above is the main idea of SVM to deal with the classification problem. At present, support vector machines have achieved good results in the application of many real problems.

RETRACTED

## 3. Comparative Experiment of PDCA Nursing Mode

### 3.1. Experimental Data

A total of 72 hospitalized children diagnosed as MPP from December 2019 to March 2020 in the 5th District of Pediatrics of the First Affiliated Hospital of Jiangxi University of Chinese Medicine were recruited and randomly divided into two groups, with 36 children in each group. All the children in the experiment were informed and approved by their guardians, and signed the relevant medical confirmation letters, which were in line with the clinical diagnostic criteria of mycoplasma pneumonia in children. Infants with mental diseases or other major diseases were strictly controlled to participate in the experiment.

Among the 36 patients in the experimental group, 18 were male and 18 were female. The age distribution ranged from 1 to 13 years, with an average age of 7.7 ± 0.1 years. The course of disease was 1 to 6 days, and the mean course of disease was 4.7 ± 0.6 days. In the control group, there were 18 male children and 18 female children. The age distribution ranged from 1 to 13 years, with an average age of 6.9 ± 0.4 years. The course of disease was 1 to 6 days, and the mean course of disease was (5.5 ± 0.3) *d*. There was no significant difference in general data between the two groups (*P* > 0.05), which was comparable.

### 3.2. Nursing Methods

The 36 children in the control group were treated with routine nursing methods. During the experiment, the nursing staff needed to check the physical conditions of the children regularly, and timely informed the doctors of any abnormal conditions in terms of the severity of symptoms, the respiratory rate and the peak expiratory value of the children, and other indicators. The 36 children in the observation group were treated with the PDCA nursing method, and different nursing structures were used in the routine nursing process. The specific PDCA nursing mode is shown in Figure 1.

1. Formulation of nursing plan: nursing staff should also take into full consideration the physical condition, family background, psychological factors, social factors, and other factors of children with mycoplasma pneumonia before making the plan. Because the nurses themselves will also have differences, which will affect the experimental effect, so before the start of the experiment, the nurses participating in the experiment should be trained uniformly, and their operation should be standardized to avoid the influence of the experimental results due to their own reasons.
2. Application of nursing plan: for children with a generally younger age, their logical awareness is low and they are unable to self-resolve their emotions. At this time, the medical staff need to stabilize the mood of the child patient according to the actual situation of the child, cooperate with playing video and music, provide the child with toys, divert the child's attention during the treatment process, reduce their pain and discomfort, and in the process of treatment, actively guide parents to cooperate with the hospital to treat their children. These nursing programs will effectively guarantee and improve the therapeutic effect.
3. The implementation of nursing evaluation: in the nursing process, a detailed nursing plan should be developed to standardize the behaviors of the nursing staff, evaluate the regular performance, and find, discuss, and solve problems in a timely manner. For children's health problems, nurses should report to the organized seminar in a timely manner, and the experts will discuss and solve them.
4. The development of nursing summary work: For the problems existing in the nursing process, the nursing staff should record, summarize, and report in time, and formulate the corresponding report uniformly after the end of the experiment. Nursing staff should also find their own shortcomings and advantages in the process of this experiment, and further improve themselves, to help children overcome the disease.

RETRACTED

### 3.3. Evaluation Index and Method

The evaluation indexes include the following: (1) the satisfaction of nursing staff in the training process; (2) time of symptom disappearance; (3) peak expiratory flow rate; (4) length of hospital stay; and (5) forced expiratory volume. Among them, in the whole nursing process, the degree of satisfaction to the nursing staff is divided into three indicators: satisfaction, basic satisfaction, and dissatisfaction. Because the children are young, they are filled in by the families of the children. The calculation formula of total satisfaction is as follows: (satisfaction + basic satisfaction)/36 × 100.00%.

Statistical Methods SPSS 24 statistical software was used for data processing. Measurement data were expressed as mean ± standard deviation, and the *χ*^2^ test was used. Enumeration data were expressed as (m, %), and the difference was statistically significant when *P* < 0.05 was used.

### 3.4. Training of Nurses

Before the start of the experiment, we conducted corresponding training for the nurses participating in the experiment, and the training period lasted for one month. As can be seen from the data collected from the training quality evaluation form, the average score for teaching objectives (full score: 10) is 9.4, and the average score for teaching attitude (full score: 10) is 9.6. The average score was 9.3, pre-class preparation (full score: 10) 8.8, blackboard writing (full score: 10) 7.7, teaching procedure (full score: 20) 18.2, and teaching effect (full score: 40) 37.2. The comparison of the average scores before PDCA quality improvement and after PDCA quality improvement is shown in Figure 2.

RETRACTED

As can be seen from Table 2, the average score of the nursing staff after quality improvement was 95, 94, 96, 9.88, and 96% in the theoretical operation examination. It can be seen that the passing rate of students has been significantly improved after the quality improvement as shown in Table 2.

## 4. Comparison and Analysis of PDCA Nursing Mode before and after

### 4.1. Satisfaction Comparison

The total nursing satisfaction of the observation group was 97.22%, which was higher than 94.44% in the control group, and the difference was statistically significant (*P* < 0.05). In the table, 21 patients were satisfied with the evaluation, which was higher than 19 patients in the control group. The PDCA nursing mode has an auxiliary effect on the treatment of mycoplasma pneumonia in children, as shown in Table 3.

### 4.2. Comparison of Hospital Stay and Symptom Disappearance Time between the Two Groups

The length of stay in the experimental group was about 12.8 days and the time of symptom disappearance was about 1.2 days, whereas the length of stay in the control group was about 12.8 days and the time of symptom disappearance was about 1.2 days. The length of stay in the experimental group was lower than that in the control group, and the differences were statistically significant (*P* < 0.05), as shown in Table 4.

### 4.3. Comparison of Peak Expiratory Velocity between the Two Groups

After active nursing, the peak expiratory velocity of the experimental group was about 43.27, which was better than that of the control group (27.12), and the difference was statistically significant (*P* < 0.05), as shown in Table 5.

### 4.4. Comparison of Treatment Time

As can be seen from Figure 3, the treatment market duration consumed by the experimental group was slightly lower than that of the control group, and the score of consumption duration was also higher than that of the control group.

As shown in Figure 3, the therapeutic market duration consumed by the experimental group was 2.93, and the duration of the control group was 3, which was slightly lower than that of the control group.

### 4.5. Comparison of Cytokine Levels

As can be seen from Figure 4, the drug residues of patients in the experimental group were higher than those in the control group, but statistically speaking, only the level of IL-2 was significantly improved.

RETRACTED

### 4.6. Comparison of Curative Effect

As shown in Table 6, the treatment effect of the experimental group was significantly better than that of the control group, and the improvement of the treatment effect was statistically significant.

### 4.7. Forced Expiratory Volume Comparison

The forced expiratory volume index of the experimental group was about 53.03, which was better than that of the control group (32.58), and the difference was statistically significant (*P* < 0.05), as shown in Table 7.

### 4.8. Nursing Staff Satisfaction Comparison

As can be seen from Table 8, not only the satisfaction of patients in the experimental group is higher than that of the control group, but also the satisfaction of nursing staff in the experimental group.

## 5. Conclusion

Mycoplasma pneumonia is a very common disease that harms the health of children. It is often clinically manifested as cough, vomiting, fever, and other symptoms. In order to further shorten the treatment time of children with mycoplasma pneumonia and help them pass through the fragile period of life, active treatment cannot be separated from good nursing plan. During the experiment, 72 children with mycoplasma pneumonia were divided into groups, and the experiment adopted the PDCA nursing model. The nursing model is divided into four stages: planning, implementation, evaluation, and summarization. The PDCA nursing model emphasizes that during the patient's recovery time, attention should be paid to taking care of the child's discomfort and problems during the nursing process. Pay attention to the children as the center of the nursing concept, and pay attention to improve the problems existing in the nursing process of children and further improve the comfort of children in the clinical nursing process. The experimental results show that in the experimental group using PDCA nursing mode, the total satisfaction is 97.22%, higher than the control group of 94.44%. In the experimental group, the hospital stay and symptom disappearance time were significantly shortened by four hours. The satisfaction of nursing staff was significantly increased in statistical significance (*P* < 0.05). Therefore, in a statistical sense, the artificial intelligence e-health PDCA nursing mode can significantly improve the clinical symptoms of MPP children with wind-heat stagnation of lung syndrome and phlegm-heat closure of lung syndrome, improve the treatment effect of childhood mycoplasma pneumonia epidemic, shorten the time of hospitalization and symptom disappeared, and play a great auxiliary role in the treatment of childhood mycoplasma pneumonia.

RETRACTED

## Figures and Tables

**Figure 1:** PDCA nursing model diagram.

**Figure 2:** Comparison of average scores before and after PDCA quality improvement.

**Figure 3:** Comparison of treatment time.

**Figure 4:** Comparison of cytokine levels.

**Table 1:** Eigenvalues and contributions of each component.

Principal component	Characteristic value	Contribution rate (%)	Cumulative contribution rate (%)
1	3.029	41.27	41.27
2	2.4481	31.84	73.11
3	1.0321	14.51	87.62
4	0.6352	7.36	94.98
5	0.3526	2.83	97.81
6	0.1568	1.82	99.63
7	0.0785	0.35	99.98
8	0.0023	0.02	100

**Table 2:** Comparison of students' test scores before and after PDCA quality improvement.

Group	Number of cases	Theory	Operation
Before quality improvement	50	82.7 ± 6	93.7 ± 2.3
Quality improvement	50	89.6 ± 3.7	95.0 ± 1.0
t		-6.89	-3.6
p		<0.05	0.001

**Table 3:** Satisfaction comparison table.

Group	Number of cases	Satisfied	Basically satisfied	Dissatisfied	Total satisfaction (%)
Control group	36	21	14	1	97.22
Observed group	36	19	15	2	94.44

**Table 4:** Comparison of hospitalization time and symptom disappearance time.

Group	Number of cases	Length of stay	Time of symptom disappearance
Control group	36	12.8 ± 2.8	1.2 ± 0.4
Observed group	36	16.5 ± 3.3	2.8 ± 2.1
T value		5.239	4.289
*P* value		<0.05	<0.05

**Table 5:** Comparison of the peak expiratory flow rate.

Group	Number of cases	Peak expiratory flow rate
Control group	36	43.29 ± 12.03
Observed group	36	27.12 ± 16.27
T value		6.178
*P* value		<0.05

**Table 6:** Comparison of curative effect between the two groups after treatment.

	The number of cases	Cure	Effective	Upturn	Invalid	Efficient (%)	*P* values
The treatment group	36	5	18	12	1	97.22	0.055
The control group	36	1	14	18	3	91.67	

**Table 7:** Comparison of forced expiratory volume.

Group	Number of cases	Forced expiratory volume
Control group	36	53.03 ± 12.53
Observed group	36	32.58 ± 12.69
T value		9.327
*P* value		<0.05

**Table 8:** Nursing staff satisfaction comparison.

Group	n	Very satisfied	Satisfied	Basically satisfied	Dissatisfied
Trained	12350	3730 (30.2)	3260 (26.4)	3433 (27.8)	1927 (15.6)
Untrained	16258	7868 (48.4)	5072 (31.2)	2243 (13.8)	1075 (6.6)
*χ*2		963.618	78.344	865.114	651.728
P		<0.001	<0.001	<0.001	<0.001

## Data Availability

No data were used to support this study.
